The article "Diagnostic Value of Susceptibility-Weighted Imaging Combined with Diffusion-Weighted Imaging in Early Intracerebral Hemorrhage" was published in 2022. Journal: Contrast Media Mol Imaging.

# Diagnostic Value of Susceptibility-Weighted Imaging Combined with Diffusion-Weighted Imaging in Early Intracerebral Hemorrhage

**DOI:** 10.1155/2022/8072582

**Published:** 2022-06-24

**Authors:** Zhanqiang Song, Junhong Peng, Xia Li, Guiping Shen

**Affiliations:** ^1^Radiology Department, Wuhan Fourth Hospital, Wuhan 430000, China; ^2^Radiology Department, General Hospital of the Central Theater Command of the PLA, Wuhan 430000, China

## Abstract

**Objective:**

The incidence of early intracerebral hemorrhage (ICH) is gradually increasing and has been shown to affect an increasing number of younger people. Conventional imaging modalities might have a low detection rate of early and small ICH lesions. This study aimed to investigate the diagnostic value of susceptibility-weighted imaging (SWI) combined with diffusion-weighted imaging (DWI) in early ICH.

**Materials and Methods:**

The data of 61 patients with early ICH diagnosed by computed tomography (CT) scan between January 2019 and February 2020 were assessed. Using CT as the gold standard, we compared the diagnostic sensitivity, accuracy, and imaging characteristics of SWI + DWI versus SWI or DWI alone.

**Results:**

A total of 78 lesions were detected by CT in 61 patients with early ICH. The diagnostic sensitivity and accuracy of SWI + DWI were significantly higher than those of SWI or DWI alone. In terms of imaging characteristics, DWI demonstrated very low signal intensity in the hematoma center at different stages of early ICH with high signal intensity in the surrounding tissue, and the signal range gradually increased over time. By contrast, SWI displayed very low signal intensity at different stages, and the signal intensity also gradually increased over time.

**Conclusion:**

Compared with SWI or DWI alone, SWI combined with DWI could improve the detection rate of hematoma lesions in patients with early ICH.

## 1. Introduction

Spontaneous intracerebral hemorrhage (ICH) refers to the spontaneous and nontraumatic rupture of blood vessels, resulting in the accumulation of blood in the brain parenchyma [1, 2]. As more blood gets accumulated, this increases the intracranial pressure, leading to neurological symptoms, such as nausea, vomiting, limb numbness, and paralysis. The incidence of ICH is gradually increasing, with 1–27 cases per 100,000 persons per year, ranking it as the second most common subtype of stroke [3]. It has a high mortality range and has recently shown a higher incidence in younger people [4]. In China, ICH accounts for 18.8%–47.6% of all cases of stroke [5]. It is an acute process characterized by dangerous pathogenic conditions, high disability and mortality, causing heavy financial and psychological burdens to families and society. Therefore, the early detection of hemorrhagic lesions and timely symptomatic treatment are important prerequisites for improving the prognosis of patients with early ICH [6].

Computed tomography (CT) is the preferred imaging examination for ICH. It can quickly and accurately display the location of hematoma and help assess the bleeding volume, spread into the ventricles or arachnoid membrane, mass effect, and damage to surrounding brain tissues. However, it also has disadvantages such as radiation exposure and unclear display of brainstem and posterior fossa lesions. Comparatively, magnetic resonance imaging (MRI) can display three-dimensional images of the brain, with advantages such as higher clarity, no exposure to radiation, and absence of skull artifacts.

Diffusion-weighted imaging (DWI) is a rapid and noninvasive MRI technique that can effectively detect hemorrhagic lesions in patients with early ICH intracerebral hemorrhage by examining the diffusion of water molecules in living tissues. Unfortunately, clinical studies have shown that the misdiagnosis rate with DWI could be high, especially in patients with neurovascular diseases, such as vascular brain tumors and cerebral infarction [7]. Susceptibility weighted imaging (SWI) is a new MRI technique based on the differences in magnetic susceptibilities of various tissues. MRI is highly sensitive to paramagnetic substances, such as hemosiderin deposition and calcium, and has a high resolution for hemorrhagic and other lesions in patients with early ICH [8, 9].

Currently, few studies have compared the clinical diagnostic reliability between DWI and SWI. In this study, we investigated the diagnostic significance of SWI combined with DWI compared with DWI and SWI alone in early ICH.

## 2. Materials and Methods

### 2.1. Patient Collection

In this study, early ICH was defined as ICH cases diagnosed on CT scans within 6 hours since the onset of signs or symptoms. Using this definition, the data of 61 patients (34 males and 27 females) diagnosed with early ICH between January 2019 and February 2020 in the Department of Neurosurgery at the Wuhan Fourth Hospital (Wuhan, China) were retrieved. All included patients were diagnosed with CT and met the diagnostic criteria of ICH according to *the Guidelines for Diagnosis and Treatment of Cerebral Hemorrhage in China* [4, 10]. Exclusion criteria were as follows: (1) time from the ICH onset to hospital admission exceeded 72 h; (2) patients who had cerebral infarction, cerebral hemangioma, and other complications; (3) patients who were transferred to another hospital for further treatments; (4) patients who had mental diseases or were unable to communicate; (5) patients who had contraindications to MRI examination; and (6) presence of a history of brain surgery, early ICH, or other cerebral diseases. All patients or their families signed informed consent forms. This study was reviewed and approved by the medical ethics committee of the Wuhan Fourth Hospital.

### 2.2. Examination Methods

The location of hemorrhagic lesions was examined using the GE discovery 3.0 T MRI scanner magnetic resonance instrument (General Electric Company, USA) 0–6 hours, 7–12 hours, and 13–24 hours after the onset. The examination sequences included SWI and DWI. Two associate chief physicians analyzed the obtained images. The specific parameters of DWI included: slice thickness = 5.0 mm, slice spacing = 1.0 mm, 6000 ms/100 ms, and *b* value = 1000 s/mm^2^. The SWI parameter settings were as follows: slice thickness = 1.2 mm, matrix = 480 × 388, TR = 36 ms, TE = 20 ms, and FOV = 20 × 24.

### 2.3. Diagnostic Sensitivity and Accuracy

Using CT examination as the gold standard and reference for ICH diagnosis, the detection rate of early ICH by DWI and SWI was estimated, and their diagnostic value in early ICH was analyzed. Sensitivity was calculated using the following formula: sensitivity = (TP/[TP + FN]) × 100%. The positive predictive value was calculated using the following equation: positive predictive value = (TP/[TP + FP]) × 100%. The accuracy of the parameters was calculated using the following formula: accuracy = ([TP + TN]/total cases] × 100%. In this study, true-positive was referred to as TP, true-negative as TN, false-positive as FP, and false-negative as FN.

### 2.4. Statistical Analysis

All statistical analyses were performed using the SPSS (version 26.0) software. Enumeration data were expressed as *n* or percentage. The chi-square test was used to compare between groups. *P* < 0.05 was considered significantly different.

## 3. Results

### 3.1. Detection of Early ICH

All patients were aged between 54 and 72 (mean ± standard deviation, 62.74 ± 4.37) years and had a body mass index (BMI) of 18–25 kg/m^2^ (21.36 ± 2.74 kg/m^2^. Among them, 44 patients had one hemorrhagic lesion, and 17 had two lesions.

Initial CT scan examinations of 61 patients identified a total of 78 ICH lesions. Using CT findings as reference, the detection rate of ICH lesions using DWI alone, SWI alone, and DWI + SWI were analyzed. Our findings showed no significant difference in positive predictive value among the three groups. However, we observed that the sensitivity and accuracy of DWI + SWI were higher than DWI or SWI alone for the detection of early ICH (Table 1).

### 3.2. Imaging Characteristics of DWI and SWI in Three Stages of Intracerebral Hemorrhage

Within 6 hours after the onset, a very low signal intensity was detected in SWI images at the center of the hematoma, which had relatively clear margins. The signal intensity of the surrounding areas was slightly higher than that of the center of the hematoma (Figure 1). Similar observations were observed on DWI images (Figure 1).

At 7–12 hours after the onset, a very low signal intensity was detected in SWI images at the center of the hematoma, which had relatively clear margins. Compared with the center of the hematoma, the signal intensity of the surrounding areas was higher. In contrast, DWI images showed that the center of the hematoma had a very low signal intensity, with transient linear hypointensity observed at the margin. Compared with the center of the hematoma, the signal intensity of the surrounding areas was higher, but although hematoma margins were clear, they started to become fuzzy (Figure 1).

At 13–24 hours after the onset, the signal intensity at the center of the hematoma was still very low on SWI images and had clear margins. However, the signal intensity of the surrounding tissues was significantly increased compared to the hematoma center. In DWI images, very low signal intensity was also detected at the center of the hematoma, but the signal intensity at the margin almost disappeared and became fuzzy. Hyperintensity could be observed in the surrounding areas of the hematoma (Figure 1).

During the onset of early ICH, both SWI and DWI were characterized by a very low signal intensity at the center of the hematoma. The signal intensity of surrounding tissues was higher than the hematoma center within the first 6 hours since the ICH onset and gradually enhanced over time. The main difference between SWI and DWI was at the hematoma margin. The signal intensity of DWI decreased from clearly visible to fuzzy from 6 hours to 24 hours after the onset, while that of SWI remained relatively clear.

## 4. Discussion

In patients with ICH, a common disease in neurosurgery, the surrounding brain tissue is compressed by hemorrhagic mass, resulting in ischemia, and hypoxia. This condition induces the release of a large number of oxygen free radicals and inflammatory factors that aggravate the damage to surrounding brain tissues and affect the prognosis of patients [11, 12]. Based on recent statistics [13], the clinical mortality rate of ICH is as high as 30%, and most of the surviving patients still present with different degrees of sequelae, such as aphasia and hemiplegia, which can severely impact the patients' quality of life. Compared with CT scans, MRI has higher tissue resolution and multisequence scanning advantages. Therefore, compared with other examination methods, MRI can detect smaller tissue lesions and provide a reliable basis for the localization and qualitative diagnosis of patients with early ICH [14].

However, conventional MRI and CT may also have some limitations. In recent years, compared with the conventional scanning sequence, magnetic SWI has been shown to offer a high signal-to-noise ratio and high spatial resolution, resulting in very high sensitivity to paramagnetic substances [15, 16]. Further, SWI has gradually started to be increasingly used in clinics by doctors because of its simplicity and convenience.

Both DWI and SWI belong to the scanning sequences of nuclear magnetic resonance. This study showed that the diagnostic sensitivity and accuracy of DWI + SWI for hemorrhagic lesions were higher than those of the two alone. DWI examination is based on the movement of water molecules and can provide information regarding the physiological state of the brain. Specifically, by applying a symmetrical gradient on either side of the 180° pulse of the spin-echo sequence, protons can be affected by gradient fields to generate different resonance frequencies at different sites, resulting in dephasing and loss of the DWI signal [17]. The pathological changes at the lesion site in patients with early ICH can inhibit Brownian motion diffusion of water molecules in the brain tissue. Thus, DWI displays abnormally a high signal intensity in the lesions and normal intensity in surrounding tissues [18]. Comparatively, SWI has a susceptibility effect on mineral elements in hemorrhagic lesions. Early ICH can cause hemosiderin deposition at the lesion, while hemoglobin at the hematoma site is converted into deoxyhemoglobin. The paramagnetic substances can produce local magnetic field changes and dephase protons, causing accelerated T2 relaxation. Therefore, hemorrhagic lesions can be sensitively diagnosed using tissue susceptibility differences [19].

This study summarized the imaging characteristics of two MRI parameters for early ICH at different time points after the onset of ICH. According to DWI images, the hematoma center displayed a very low signal intensity with higher signal intensity in surrounding tissues, which gradually increases over time. In contrast, SWI images showed that the hematoma center also displays a very low signal intensity at different time points after the onset, and the signal intensity at the margin gradually increases over time. The reason for such results of DWI imaging could be due to changes in the molecular structure of hemoglobin and contraction of intact red blood cells leading to a reduction of intracellular space and low signal intensity in the center of the hematoma, while perihematomal tissues present a hyperintense state due to the change in blood concentration and its degradation products, as well as vasogenic edema caused by disruptions in the blood-brain barrier. In addition, at 7–12 h after the ICH onset, a transient linear hypointensity at the edge of the hematoma could be observed from DWI images, which could be associated with artifacts produced by oxygen exchange between perihematomal red blood cells and surrounding tissues, resulting in the water molecule movement [20, 21]. Patients with early ICH have uniform magnetic fields attributed to the paramagnetic susceptibility of deoxygenated hemoglobin, causing different proton spin frequencies in surrounding tissues and forming a phase difference. As a result, tissues with different magnetic sensitivity can be distinguished on the SWI phase diagram. After further image processing, the original phase diagram and magnitude image can be combined to form a new magnitude image, leading to maximized contrast and magnetic sensitivity difference between the hematoma and normal tissue. As hemoglobin deoxygenation at the hematoma becomes more evident over time, leading to a greater paramagnetic difference between the lesion and surrounding tissues, and higher SWI signal intensity [22–24].

It is also worth noting that in this study, the detection rate of SWI combined with DWI for early ICH was 100%, which was comparable to that of CT. In addition to the high detection rate, SWI combined with DWI could overcome the disadvantages of CT, such as exposure to radiation and skull artifacts [25]. Further, it has also been shown that on some occasions, compared to CT scans, SWI MRI sequences could improve the detection of smaller lesions, which could be found during early ICH [16, 26]. Therefore, the combined examination using SWI and DWI could be an alternative for patients unsuitable for CT, such as pregnant women and others, or those with small early lesions.

## 5. Conclusion

In summary, our findings showed that SWI combined with DWI demonstrated comparable detection rates with CT scans but had a higher diagnostic value than SWI alone and DWI alone for early ICH diagnosis in Chinese patients. This could provide an alternative for early detection of smaller lesions or assessment of patients unsuitable for CT scans, but these findings should be validated in larger cohorts of patients using prospective and randomized settings before clinical application.

## Figures and Tables

**Figure 1:** Image characteristics of DWI and SWI at three different periods since intracerebral hemorrhage the onset. DWI, diffusion-weighted imaging; SWI, susceptibility-weighted imaging.

**Table 1:** Detection of early intracerebral hemorrhage based on three MRI parameters.

Parameters	Detected hemorrhagic lesions (*n*)	Sensitivity	Positive predictive value	Accuracy
DWI	72	92.30 (72/78)	100.00 (72/72)	92.30 (72/78)
SWI	74	94.87 (74/78)	100.00 (74/74)	94.87 (74/78)
DWI + SWI	78	100 (78/78)^*∗*^^#^	100.00 (78/78)	100 (78/78)^*∗*^^#^

Note.^*∗*^*P* < 0.05*vs*. DWI; #*P* < 0.05 *vs*. SWI; DWI, diffusion-weighted imaging; SWI, susceptibility-weighted imaging.

## Data Availability

The data used to support the findings of this study are available from the corresponding author upon request.
